The article "Maintenance and Management Technology of Medical Imaging Equipment Based on Deep Learning" was retracted in 2023. Reasons: unreliable results or conclusions; concerns about the data; concerns about the peer review; concerns about the citations.

# Maintenance and Management Technology of Medical Imaging Equipment Based on Deep Learning

**DOI:** 10.1155/2022/6361098

**Published:** 2022-07-01

**Authors:** Bin Liu, Lingli Tong, Yanmei Liu, Zhizhang Guo

**Affiliations:** Shandong Provincial Hospital Affiliated to Shandong First Medical University, Shandong, Jinan 250021, China

## Abstract

Medical equipment maintenance in modern hospital management is an emerging marginal discipline which is one of the important branches of hospital management with the dual function of management and technology. The good or bad management of medical equipment directly affects the quality of hospital work. With the development of science and technology, the scale of hospitals continues to expand and develop; hospitals are equipped with more and more medical equipment and its technical content is getting higher and higher, which makes the medical equipment management and maintenance practitioners more demanding. However, the situation of existing medical equipment management and maintenance personnel is not optimistic. For this reason, this paper designs a good database structure, which can effectively reduce data redundancy and better avoid the problems that may occur during the database operation. As a reference guideline for database design, the three database paradigms can be studied and understood in depth to help software designers design more “robust” databases, enabling effective maintenance and management of medical imaging equipment.

## 1. Introduction

As the trend of engineering, intelligence, and networking of medical diagnosis and treatment technology becomes more and more obvious, the proportion of medical equipment in medical and health care expenditure is also increasing [1]. The personnel engaged in medical equipment management and maintenance should also be improved year by year and the quality requirements of these personnel are getting higher and higher, but the actual situation is that their status in the hospital is not clear, they are mostly under the auxiliary departments or logistics departments, and the trend of being weakened and marginalized weakened the role of medical equipment management and maintenance in the overall medical activities [2]. Some hospitals even cancel the medical equipment management department to engage in the marketization and socialization of medical equipment maintenance, which makes medical equipment management and maintenance can not meet the clinical needs in terms of timeliness or economy, resulting in a shortage of medical equipment management and maintenance personnel and a large number of job-hopping; many people have switched to become agents of major foreign medical equipment companies [3].

The article "Maintenance and Management Technology of Medical Imaging Equipment Based on Deep Learning" was retracted in 2023. Reasons: unreliable results or conclusions; concerns about the data; concerns about the peer review; concerns about the citations.

As the degree of integration increases, the complexity of the equipment also increases, while the localization rate of medical equipment is not high, so we are limited in the field of medical equipment [4, 5]. Technology is monopolized coupled with large equipment by the manufacturer's warranty, does not provide drawings, sets the password, maintenance technology blockade, and so on, and causes the rate of self-repair of equipment to decline. Especially for some high-grade precision equipment to buy a warranty has become a trend. Medical equipment maintenance surface is increasingly narrow plus a variety of different types of equipment whose professional division is too fine; existing technical personnel can only solve some basic maintenance of equipment [6]. Due to the obvious lack of technical personnel, many people are working in several jobs; it is difficult to do fine and is specialized also in making medical equipment management and maintenance personnel work under increased pressure; in addition, relatively low treatment promotion is hopeless; career prospects are generally not favored [7–9].

## 2. Related Work

In order to achieve more and better research results in the field of imaging using deep learning techniques and put them into clinical applications as early as possible, based on the model and characteristics of deep learning, researchers are first required to have a large amount of medical image annotation data, while a traditional manual annotation is too time-consuming and laborious, the accuracy of automatic annotation [10] is not yet up to the requirement of deep learning techniques for high accuracy of datasets, and the results are annotated by traditional methods. The traditional medical image annotation methods and results are therefore not suitable for use in deep learning research methods [11]. In terms of medical image annotation tools, although there are many software systems for medical image processing from well-known large companies in the medical field, such as Neusoft Medical, Heiner Medizin, and Siemens at home and abroad, no company or enterprise has yet developed a perfect annotation system for deep learning technology in medical image annotation as a new research hotspot combined with the field of imaging. Although some image annotation widgets exist, they all have a single function and do not have the functions of acquiring medical big data, data storage, data statistics, annotation of many types and formats of medical images, and their visualization [12]. Therefore, how to extract a large number of different kinds of medical image data from different hospital PACS system databases, store, manage, report, browse, and annotate the images and annotation file formats that can be directly used for deep learning, and then provide a large number of databases for the research progress of deep learning technology in the medical field is the primary problem that is commonly faced and urgently needed to be solved by experts and scholars who apply deep learning technology to the medical field [13–18].

The article "Maintenance and Management Technology of Medical Imaging Equipment Based on Deep Learning" was retracted in 2023. Reasons: unreliable results or conclusions; concerns about the data; concerns about the peer review; concerns about the citations.

## 3. Overall System Design

### 3.1. Overall Architecture Design

Based on the research at the hospital site and the analysis of the current needs in the field of medical image research, the design of this project divides the overall system architecture into the following three levels: interface layer, functional layer, and data exchange layer, as shown in Figure 1. As the name implies, the interface layer is the common system operation interface, which can be seen directly by the user when starting the software system [19]. The design of the interface layer generally follows the following principles: to ensure the perfection of the functions while making full use of the interface space, consistent background color, neat typography, different font sizes, and prominent functional modules, so that the interface looks beautiful and generous as a whole, comfortable for the user to use, and easy to operate; the functional layer is mainly used to receive and implement requests for various functions on the interface, and to minimize the overall. The data exchange layer is mainly used to complete the data connection and exchange between the database and the client, which is responsible for the data exchange between the whole system and the database, and the design of the data exchange layer needs to comply with the following principles: to ensure that the system can connect to the requested database when needed and perform common database operations such as adding, deleting, changing, and checking the corresponding database table data, and to require that the system can be connected to the database when needed. It is also required that the operation process should not affect other database table data and be accurate [20].

### 3.2. Database Design

A well-designed database structure can effectively reduce data redundancy and better avoid possible problems during database operations. As a reference guideline for database design, an in-depth study and understanding of the three paradigms can help software designers to design a more “robust” database.

Based on this, the database table design in this project strictly follows the basic principles of the three paradigms.

*The First Paradigm (1NF)*. Atomicity, as a typical feature of the first paradigm, determines that each field in a database table is a single attribute and cannot be subdivided; i.e., no more than one value can appear in the same column, as shown in Table 1, which satisfies this paradigm, and Table 2, which does not satisfy this paradigm.

The article "Maintenance and Management Technology of Medical Imaging Equipment Based on Deep Learning" was retracted in 2023. Reasons: unreliable results or conclusions; concerns about the data; concerns about the peer review; concerns about the citations.

*The Second Paradigm (2NF)*. The second paradigm is based on the first paradigm, which means that the second paradigm is satisfied only if the first paradigm is satisfied first. The column used as the unique identifier for each instance in this paradigm table is called the primary key or primary keyword. This column with a unique identifier ensures the uniqueness of the data rows in the table and avoids the situation where some field values will depend on some of the fields to exist, thus doing away with partial dependencies. If, because there are multiple primary keys in the table, some of the fields are completely dependent on the primary key, while the rest of the fields are partially dependent on one of the primary keys, the situation of partial dependency will arise. At this time, in order to make the table structure conform to the second paradigm, we split the table and use the split primary key as the unique primary key of each new table, respectively, so that the new tables all become fully dependent, which can satisfy the second paradigm.

*The Third Paradigm (3NF).* Satisfying the third paradigm presupposes that the second paradigm is satisfied first. This paradigm requires that all fields in the table other than the primary key depend directly on the primary key, and there can be no passing dependencies. By passing dependency, we mean that nonprimary key column 1 depends on nonprimary key column 2, while nonprimary key column 2 depends on the primary key. Since the fields that generate pass dependency are redundant fields, the design of the third paradigm eliminates the pass dependency while better avoiding data redundancy. Similar to the second paradigm, when a pass dependency occurs, it can also be solved by using relational decomposition, where the field in the original table where the pass dependency occurs is taken out and put into a new table, and the primary key of the new table is set to the dependent field in the original table, at which time the field is treated as a foreign key of the original table.

According to the design architecture of the whole system, the database relationship diagrams used for each functional module are drawn separately using the entity-connection diagram as shown in Figure 2.

As shown in Figures 3–5, the database tables of each module are designed according to the relationship diagram; the patient information table to save the migrated data, the Bucket table to manage the cloud storage files, and the annotation table to manage and save the information related to the data to be annotated and annotated, etc., are created, respectively.

The article "Maintenance and Management Technology of Medical Imaging Equipment Based on Deep Learning" was retracted in 2023. Reasons: unreliable results or conclusions; concerns about the data; concerns about the peer review; concerns about the citations.

The first step is to design the database tables for the data migration module. The database table of this module contains the record and storage of basic information about patients, examination, and diagnosis report information and examination and diagnosis image information. According to the field research, in order to meet the demand of each department for patient information, the basic information of patients, examination and diagnosis reports, and image information are usually stored in different database tables, so for the operation process of this system, if the basic information of patients and diagnosis reports and image information are also stored in different database tables when designing.

Finally, the database table of the image annotation module is designed to record and store the image files and XML files generated after the annotation, as well as the information of each annotated patient. The fields in the annotation information table mainly include ImaNum, XmlNum, AnnotationDoctor, AnnotationFlag, DicomPath, XmlPath, PNGPath, path (PngPath), and other basic patient information corresponding to this data. Among them, the image number and XML file number are the primary keys of the table, which represent the unique numbers of the saved images and generated XML files after annotation, and are automatically generated during the annotation process, and the two numbers correspond to each other; since the whole annotation process requires the participation of at least three expert physicians, the annotation expert field is used to record the annotation physicians of each data. The DICOM file path, XML file path, and PNG file path are used to record the location where each image data is saved on the server after annotation. [21–23]

### 3.3. Data Exchange Layer Design

The data exchange layer is responsible for the connection between the system and the database and the system's operation on the database, which is designed to be implemented through ADO (ActiveX Data Objects). As an object-oriented programming interface, it is not only a powerful programming model for data access but also the simplest, most direct, and efficient way to manipulate the databases currently supported by Microsoft. In addition, this method provides a lot of convenience for programmers due to its ease of use, speed, low memory consumption, and other advantages.

ADO (ActiveX Data Objects) contains the following objects: Connection, Command, Field, Parameter, Record, Recordset, Property, Error, Stream, and so on. Error, Stream objects, etc. The object model is shown in Figure 6.

The article "Maintenance and Management Technology of Medical Imaging Equipment Based on Deep Learning" was retracted in 2023. Reasons: unreliable results or conclusions; concerns about the data; concerns about the peer review; concerns about the citations.

The specific steps of using ADO to operate the database are as follows:

1. First, add a reference to the ADO dynamic library file and initialize the library environment
2. Second, connect the system to the database through the Connection object
3. Then, the corresponding SQL statement is operated by the Command object, and the data set of the execution result is obtained by the Recordset object
4. Finally, the database connection is disconnected and the corresponding objects are released

The DataManager class in the program design contains the operations related to the whole system and the database. The SqlConnection object for establishing database connection is created in the constructor of the DataManager class, and the configuration information in the set.ini configuration file is read, including the IP address of the specified database, the name of the database, the database user name, and the database login password, to connect to the specified database. The main functions contained in the DataManager class are RunSqlCommand, GetDS, etc. Among them, the Run SQL Command function is mainly responsible for executing the SQL statements passed as parameters in the database connected to the program, more commonly used to execute database update and delete statements, etc.; the main function of the Get DS function is to obtain the information stored in the database in the form of data sets. It is mainly used when the system performs query operations. First, edit the corresponding SQL statement; second, create a new DataManager class object; second, import the SQL statement to be executed into the corresponding function; finally, use the function executed by the object to realize the operation of the specified database information.

## 4. Maintenance of Medical Imaging Equipment

Medical imaging equipment is a large and valuable piece of precision medical equipment, especially X-ray imaging means such as CR, CT, and other imaging pieces of equipment. With the development of science and technology, medical imaging equipment has developed into a set of computers, electronics, mechanical optics, materials science and other technologies, complex structure, a wide range of functions, and high prices of large expensive precision medical equipment. In clinical applications ensuring that the imaging equipment is in good condition is the basis for the accuracy of patient diagnosis; therefore, it is very important to strengthen the daily maintenance of imaging equipment. The maintenance of medical imaging equipment includes proper use, daily maintenance, and a regular overhaul.

The article "Maintenance and Management Technology of Medical Imaging Equipment Based on Deep Learning" was retracted in 2023. Reasons: unreliable results or conclusions; concerns about the data; concerns about the peer review; concerns about the citations.

### 4.1. Compliance with Operating Procedures

In order to ensure the normal operation of CR and CT, a set of operating procedures are arranged according to their structure and performance characteristics. Due to the differences in the structure of the equipment, the operating procedures are not the same. The operating procedures are generally as follows:

1. Before operating the equipment, first of all, we should first check whether the console instruments switch in the normal position [24–26].
2. Turn on the power switch, power on, and the equipment is in the warm-up process.
3. According to the specific needs of fluoroscopy or camera, select the appropriate technical parameters. In the selection of camera exposure conditions should pay attention to the m A, kV, and exposure time selection order; we generally should first choose the m A value, then choose the kV value, and do not first choose the kV value, after the m A value.
4. In the operation of the foot control switch or a manual switch, the action should be rapid, and the force should be balanced and appropriate.
5. Finish using the equipment, turn off the machine, set the regulator to the lowest position, and finally turn off the main power supply.

### 4.2. Routine Maintenance of Medical Imaging Equipment

Daily maintenance work includes careful operation, keeping the machine room dry, good cleaning and hygiene, paying attention to safety inspection, and other aspects.

Preventing excessive force and strong vibration, especially X-ray tube, spot film frame, etc., should be more careful when moving to prevent damage to X-ray tube and other precision fragile devices due to collision.

### 4.3. Doing a Good Job of Cleaning and Sanitation to Keep the Equipment Clean

Preventing dust from entering the interior of the equipment is an important part of daily maintenance. Entering dust into the interior of the equipment for a long time, but not removed, will make some components have poor contact, such as poor contact between the relay contacts, etc., and also make some components have short circuits, such as autotransformer interturn short circuit. Adhere to the daily work and first clean the equipment and indoor treatment. Dust removal is best to use a dust collector and try not to use a wet cloth to wipe [27–29].

*Antivibration*. X-ray tubes in transport and use should pay special attention to antivibration and antitouch. As the anode is heavy and work anode will generate a lot of heat, so transport and use should be flat or let the anode face down.

*Attention to the Exposure Interval*. X-ray machines in the continuous work should be necessary intervals to make cooling and the surface temperature of the tube sleeve more than 50–60°C.

The article "Maintenance and Management Technology of Medical Imaging Equipment Based on Deep Learning" was retracted in 2023. Reasons: unreliable results or conclusions; concerns about the data; concerns about the peer review; concerns about the citations.

*Observation Window*. X-ray tube sleeve maintains a sufficient amount of insulating oil, often through the window to observe whether the tube sleeve Air bubbles exist and if there should be timely replenishment of oil exhaust. Observe whether the X-ray tube focuses on the center of the window; otherwise, it will affect the results of photography.

*Glow*. The exposure, such as an X-ray tube, emits a very faint glow, due to some electron impact on the glass wall. The outline of the fluorescence must be distinguished from the ionization discharge phenomenon that occurs due to poor vacuum. The former occurs in the glass wall; kV increases and weakens; the latter increases with kV and is enhanced. The weak fluorescence of the glass tube wall does not affect the normal use of the X-ray tube. However, a mild glow discharge is a precursor to X-ray tube damage.

Listen to the sound: when the high voltage occurs, if there is a discharge sound, it should immediately stop working and repair [30].

## 5. System Applications

### 5.1. Operation Parameter Monitoring

The system provides real-time monitoring of the operating parameters of the important components of the equipment, including the number of exposures of the bulb, bulb temperature, cooling oil temperature, liquid helium level and pressure, cold head temperature, temperature, and humidity of the machine room. It also sets up thresholds and notifies the equipment security personnel in time if the thresholds are exceeded. The following is a description of several important monitoring parameters.

#### 5.1.1. CT Bulb Tube Temperature

The spherical tube is one of the core components of CT, which consists of a tube core, tube sleeve, and supporting oil circulation cooling system, where the tube core includes a rotating anode, cathode, and rotating shaft bearing. When the cathode electron beam bombards the focal point on the anode target surface, about 99% of the heat energy and 1% of the ray energy will be generated, so the spherical tube will generate a lot of heat. Once the bulb overheats, it can lead to high voltage fires, filament volatilization, and other malfunction phenomena. Therefore, real-time monitoring of the tube temperature and the correct and reasonable use of the tube not only can obtain high-quality images but also can extend the life of the tube (Figure 7).

#### 5.1.2. Scanning Rack Temperature

X-ray exposure will generate a lot of heat, due to the vacuum environment inside the core and heat in the form of radiation to the outer wall of the core, through the cooling of oil to absorb heat; cooling oil is cooled by the radiator. Scanning rack temperature can reflect the bulb tube cooling, thermal efficiency, most CT high load operating hours, the scanning rack temperature of 32∼36°C, and the scanning rack alarm temperature of 40°C; see Figure 2.

The article "Maintenance and Management Technology of Medical Imaging Equipment Based on Deep Learning" was retracted in 2023. Reasons: unreliable results or conclusions; concerns about the data; concerns about the peer review; concerns about the citations.

#### 5.1.3. Liquid Helium Levels and Pressures

The magnetic field of a superconducting type magnet is established by passing current to the superconducting coil in a superconducting environment to generate a strong magnetic field [14]. Maintaining a strong magnetic field for a long time is required to keep the superconducting coil in an ultralow temperature environment (superconducting coil operating temperature of 4.2 K). Maintaining an ultralow temperature environment requires liquid helium as a refrigerant, and the superconducting coil is immersed in a container filled with liquid helium. Under normal conditions, the liquid helium pressure ranges from 3.8 to 4.2 psi (1 psi = 6.89476 kPa) and the liquid helium capacity should be greater than 60% (50% is the limit). If the liquid helium pressure exceeds the normal value or if the liquid helium capacity is less than the limit value, there is a risk of loss of excess (Figure 8).

#### 5.1.4. Machine Room Temperature and Humidity

Under normal circumstances, the scanning room temperature should be controlled at 20∼25°C; too high and too low temperatures will affect the uniformity and stability of the magnet temperature center frequency, which will also lead to the magnet temperature control system not to work properly. Scanning room humidity is generally controlled at about 50% to 60%; too high humidity will cause the gradual oxidation and corrosion of components; too low humidity will cause an electrostatic phenomenon, resulting in the fact that a large amount of dust adsorption can not dissipate heat, causing a crash.

### 5.2. Remote Troubleshooting

By establishing a fault diagnosis database, when the system acquires fault codes, the best confidence solution is matched from the database by a hybrid algorithm based on constraints and division association rules and fed back to the engineer. The database is used to store the knowledge related to the repair and maintenance of imaging equipment and its corresponding set of fault phenomena, which comes from expert experience, maintenance manuals, existing knowledge related to imaging equipment, and knowledge mined from logs, and through log mining, association rules between faults are generated and updated into the fault diagnosis data.  Table 3 shows the 3.0 T MRI remote fault diagnosis table of our hospital.

### 5.3. Fine Management of Operation and Use

Real-time statistics show the number of daily scans, scanning time, number of examinations, scanning mode and parts, etc., and generate monthly reports in PDF format. The report is mainly divided into two parts; the first part is through a comprehensive analysis of monthly scanning data and dynamic comparison with historical data, from the operational efficiency of each part of the decision indicators for in-depth analysis, multiangle display imaging equipment monthly workload, and equipment usage. The second part is a comprehensive analysis of the operating data of the equipment, including a comprehensive analysis of the monthly scanning calendar, scanning volume distribution, scanning time distribution, utilization rate and scanning efficiency, scanning coils and scanning parts, and a multifaceted, multiangle comparison and display of the operating efficiency of the equipment.

The article "Maintenance and Management Technology of Medical Imaging Equipment Based on Deep Learning" was retracted in 2023. Reasons: unreliable results or conclusions; concerns about the data; concerns about the peer review; concerns about the citations.

## 6. Conclusions

The best maintenance of the correct use of medical imaging equipment, good routine, and regular maintenance of medical imaging equipment can avoid most of the failures, greatly extending the life of the equipment; a well-designed database structure can effectively reduce data redundancy and better avoid the database operation process and problems may appear. As a reference guide for database design, three database examples can be studied and understood in depth to help software designers design a more “robust” database. There should be effective maintenance and management of medical imaging equipment. Engineers engaged in overhaul work should have the appropriate professional knowledge and certain work experience; overhaul should be done well in advance and then in accordance with the plan to do a good job in advance of the overhaul plan, and then gradually check according to the plan to avoid “blind” overhaul without a plan and overhaul tool specifications to complete, disassemble the wire to number, and disassemble the screws and nuts to be placed in a safe location; pay attention to their own effective protection and maintenance and equipment, and damaged parts should be replaced in a timely manner.

## Figures and Tables

**Figure 1:** Schematic diagram of the entire system architecture.

**Figure 2:** Data migration module of the entity-linkage diagram.

**Figure 3:** Entity-linkage diagram of the data storage module.

**Figure 4:** Entity-linkage diagram of data statistics module.

**Figure 5:** Entity-linkage diagram of the data annotation module.

**Figure 6:** Schematic diagram of the ADO object model.

**Figure 7:** CT bulb tube temperature and scan frame temperature profile.

**Figure 8:** MR liquid helium level and pressure profile.

**Table 1:** Example of the first paradigm.

Field	2	3	4
Data	2	3	4

**Table 2:** Example of not satisfying the first paradigm.

Field	2	3		4
Data	2	3.1	3.2	4

The article "Maintenance and Management Technology of Medical Imaging Equipment Based on Deep Learning" was retracted in 2023. Reasons: unreliable results or conclusions; concerns about the data; concerns about the peer review; concerns about the citations.

**Table 3:** 3.0 T MR remote troubleshooting table.

2019.9.15 08:00:03	Risk	The communication error of the sickbed drawing motor occurred twice on September 14, 2019	Restart after a major shutdown and replace PHPs or Sri
2019.09.15 08:00:03	Risk	The resistance value of gradient coolant is low, which occurred twice on September 14, 2019	Gradient water-cooled degasser treatment or addition of deionized water
2019.09.15 08:00:04	Risk	HEC detected that the pressure of the gradient water cooling pipeline was too low, which occurred twice on September 14, 201909	Check gradient coolant shutdown and restart

## Data Availability

The experimental data used to support the findings of this study are available from the corresponding author upon request.
